# Emerging therapies and recent advances for Tourette syndrome

**DOI:** 10.1016/j.heliyon.2023.e12874

**Published:** 2023-01-07

**Authors:** Chih-Yi Chou, Julian Agin-Liebes, Sheng-Han Kuo

**Affiliations:** a Department of Neurology, College of Physicians and Surgeons, Columbia University, New York, NY, USA; b Initiative for Columbia Ataxia and Tremor, Columbia University, New York, NY, USA

**Keywords:** Tourette syndrome, Tics, CBIT, rTMS, Neurofeedback, DBS, GPi, CM-Pf, SLITRK, CELSR3

## Abstract

Tourette syndrome is the most prevalent hyperkinetic movement disorder in children and can be highly disabling. While the pathomechanism of Tourette syndrome remains largely obscure, recent studies have greatly improved our knowledge about this disease, providing a new perspective in our understanding of this condition. Advances in electrophysiology and neuroimaging have elucidated that there is a reduction in frontal cortical volume and reduction of long rage connectivity to the frontal lobe from other parts of the brain. Several genes have also been identified to be associated with Tourette syndrome. Treatment of Tourette syndrome requires a multidisciplinary approach which includes behavioral and pharmacological therapy. In severe cases surgical therapy with deep brain stimulation may be warranted, though the optimal location for stimulation is still being investigated. Studies on alternative therapies including traditional Chinese medicine and neuromodulation, such as transcranial magnetic stimulation have shown promising results, but still are being used in an experimental basis. Several new therapies have also recently been tested in clinical trials. This review provides an overview of the latest findings with regards to genetics and neuroimaging for Tourette syndrome as well as an update on advanced therapeutics.

## 1 Introduction

Tourette syndrome (TS) is a heterogenous disorder that affects individuals of all ages worldwide and does not have a cure. The primary clinical features of TS are tics, which are varied in their phenomenology and severity and typically have co-morbid psychological conditions. Currently, the Food and Drug Administration (FDA) approved medications are pimozide, haloperidol and aripiprazole; however, extrapyramidal side effects still limit their use [1]. Behavior therapy remains first line treatment for TS [2,3]. Recent advances in genetics, neuroimaging and electrophysiology have dramatically improved our understanding of TS. This review aims to highlight the latest therapeutic developments for TS as well as new discoveries in TS pathophysiology and genetics.

## 2 Epidemiology

TS affects between 0.3% and 1% of the general population [4]. The age of onset for TS is typically between the ages of 5–6 years old, and the disease severity usually peaks at 10–12 years old with some obtaining complete remission by adulthood [5]. The prevalence of TS is higher in boys at diagnosis, however despite the higher prevalence in boys, TS is more persistent in girls [6]. The severity of TS peaks at a later age for girls than boys and the remission with age is less likely in girls [7]. One particular study of 53 people with TS found that only 63.6% of women experienced a decrease in tic severity (compared to the 88% of men) while only 1 (9.0%) woman reported a complete remission of her tics (compared to the 38.0% of men) [7]. Studies suggest that these discrepancies may be due to differences in hormones between girls and boys. More children with TS are born to mothers with higher levels of androgens while estrogen has been found to ameliorate pre-menstrual tics [8,9]. Eighty-five percent of individuals with TS can also have other neuropsychiatric comorbidities, such as attention deficit hyperactivity disorder (ADHD) and obsessive-compulsive disorder (OCD) with a gender disparity noted in these comorbidities. Specifically, ADHD is more common in boys with TS than girls with TS (58.5% *vs.* 42.3%; *p* < 0.01); on the other hand, OCD is more common in girls with TS than boys with TS (57.1% *vs*. 47.5%; *p* < 0.01) [10]. Girls with TS, when compared to boys with TS, are also more likely to have anxiety (48.0%% *vs.* 32.0%; *p* < 0.001) and eating disorders (7.0% *vs* 0.3%; *p* < 0.001) [10].

In the United States, there is a higher prevalence of TS in non-Hispanic whites (0.29%) compared to Hispanics (0.10%) and African Americans (0.04%) [11]. Interestingly, there seems to be a higher prevalence in Asian populations. TS prevalence is around 0.56% in Taiwan and 0.40% in Hong Kong; however, there has not been an update of TS epidemiology for several years in these areas [12,13]. More recent studies found that tic disorder prevalence rate in is 0.29% in Korea, but there have been no studies about TS [14]. The tic disorder prevalence is 6.1% in China with a TS prevalence of 0.3% [15].

### 2.1 Clinical features of Tourette syndrome

The core clinical features of TS are tics, which has a unique phenomenology. Tics are involuntary or semi-involuntary, sudden, brief, intermittent, repetitive movements (motor) or sounds (phonic) and often stereotypical. Tics can be categorized into simple tics, which involve a single muscle or group of muscles, or complex tics, which are more coordinated movements of a motor sequence. Motor tics are repetitive non-rhythmic movements such as eye blinking, head jerking, kicking and jumping. Phonic tics are repetitive movements involving respiratory muscles resulting in audible sounds such as sniffing, coughing and cursing [16]. Complex tics can be presented as copropraxia (obscene gestures) or echopraxia (imitating another's gestures), which are often considered socially inappropriate movements. There is often a premonitory urge preceding a tic. During this urge period, many patients report sensory symptoms such as paresthesias or dysesthesias in their body parts, which can also manifest as tickling or discomfort prior to the tics. Tics are often transiently suppressible; however, this could lead to a build-up of such an urge and result in a rebound phenomenon with bursts of tics. After a tic happens, individuals may feel a sense of relief. Therefore, tics are sometimes considered semi-involuntary movements with sensory components.

### 2.2 Diagnosing Tourette syndrome

The diagnosis of TS comes from either the Diagnostic and Statistical Manual of Mental Disorders 5th edition (DSM-5) or the International Classification of Disease (ICD-11). The DSM-5 classifies TS as a spectrum of tic disorders with TS being the most severe. In the ICD-11, TS was removed from the category of emotional disorders and classified as a movement disorder [4]. Both criteria require the presence of multiple motor tics and at least one phonic tic (though not necessarily concurrently) for 12 months and onset before the age of 18. Tics must occur multiple times a day and almost every day with no tic-free phase exceeding three consecutive months. The etiology of the tics must not be a direct effect of any substance like cocaine or other medical conditions such as Huntington's disease [17]. According to the DSM-5, TS is the most common cause of tics, though tics can occur in secondary tourettism, which can be due to infections, toxins, brain injuries, or tumors [18]. Differentiation of TS from secondary tourettism can be challenging as it requires ruling out other diseases before reaching the diagnosis of TS [18]. For those who do not have persistent tics, they have what is known as a transient tic disorder. As the name suggests, a transient tic disorder is temporary, with symptoms lasting less than a year cumulatively [16,17]. For those with pure motor tics or pure phonic tics (not both) they are considered to have persistent or chronic tic disorders rather than TS [17].

### 2.3 Tourette syndrome rating scales

Rating scales have been developed to measure the severity of tics for clinical monitoring and research. The Yale Global Tic Severity Scale (YGTSS) is the most commonly used scale in recent clinical trials [19]. The YGTSS consists of an interview, a questionnaire, and a self-rated impairment scale. The questionnaire has individuals self-evaluate which types of tics they exhibit with a motor tic checklist and a phonic tic checklist. Then the questionnaire asked the individuals to rate the severity of their tics taking into account the number of tics, frequency, intensity, complexity, and interference [20]. The impairment scale rates the impact of said tics on their day-to-day life [20]. The YGTSS score consists of domain scores: total motor tic score (0-25), total verbal tic score (0-25), total tic score (0-50), overall impairment rating, and global severity score (0–100). Total tic score is the sum of the individual motor and verbal tic scores. A higher score corresponds to more severe tics [21]. In 2021, a study evaluated 706 TS children and adolescents to study the reliability of the YGTSS, and found that the YGTSS correlates well with the Clinical Global Impression Scale for tics, but has low or medium correlations with clinical severity ratings for ADHD and OCD, demonstrating that the YGTSS is specific for tics [22].

### 2.4 Current treatments and therapy options

Therapeutic interventions for TS involve a multi-disciplinary approach that includes pharmacological, behavioral, and in severe cases, surgical approaches. Behavioral therapy is considered first-line therapy for TS [2]. Behavioral therapy aims to improve tic symptoms through habitual conditioning [23]. Patients with TS are trained to recognize premonitory urges and practice methods to voluntarily suppress tics during the urge period [24]. For TS, psychoeducation is important but not enough to treat tics alone. It can serve as a bridge from diagnosis to acceptance of treatment and can help to treat co-existing neurological disorders or psychiatric disorders [23,25]. The main form of behavioral therapy recommended to treat TS is Comprehensive Behavioral Intervention for Tics (CBIT), which is mainly Habit Reversal Training (HRT). This is recommended by the European clinical guidelines, Canadian guidelines, and American Academy of Neurology (AAN) [2,26,27]. Exposure and Response Prevention (ERP) is also another form of behavioral therapy but not as commonly used. HRT involves training a patient to recognize premonitory urges for each kind of tic that the patient exhibits and then implement a response which prevents that specific tic from occurring [28]. CBIT can be implemented in addition to HRT and can help prepare TS patients in cases where tics occur unexpectedly or help the patient identify triggers for tics [28].

Pharmacological therapy is another option for patients with TS and is frequently used in conjunction with behavior therapy. D2 blocking agents are among the most effective therapies for TS [29], and the commonly used D2 blocking agents are aripiprazole, fluphenazine, haloperidol, olanzapine, pimozide, and risperidone [30,31]. These agents can provide symptomatic benefit, but the long-term use of D2 blocking agents can be associated with side effects such as tardive dyskinesia, which may limit their use. Alpha-2 adrenergic agonists such as clonidine and guanfacine tend to be weaker but well-tolerated choices for TS [30]. Topiramate, a glutamate receptor antagonist, has been shown to be effective in treating TS [32,33]. Tetrabenazine, a vesicular monoamine transporter type 2 (VMAT2) inhibitor that depletes dopamine from the synaptic terminals, can also be used for TS; however, tetrabenazine can be associated with adverse effects, including nausea, drug-induced parkinsonism, and depression [[34], [35], [36]]. Benzodiazepines, such as clonazepam, can be effective for mild TS. Baclofen may be beneficial for children with TS though a study has found that baclofen does not necessarily reduce tics but rather improves children's sense of well-being [37].

Deep brain stimulation (DBS) is an invasive treatment that is reserved for severe cases that do not respond to other treatment methods [38]. This will be discussed further in a later section.

Exercise has shown promise as a therapy for children and adults with mental health disorders and has also been investigated for TS. Reilly et al. reviewed seven studies looking at the effect of exercise on children with TS and found that there is some evidence for reduction in tic severity and frequency, but are unable to conclude if there is any impact on TS comorbidities such as OCD and ADHD [39]. Unfortunately, these benefits may not be sustained as the studies which had follow up of the participants found that tic improvement had ceased [40,41]. Longer term studies are needed to further elucidate the exercise effects in TS.

### 2.5 Recent clinical trials

Due to limited treatment options for TS, novel pharmaceutical agents, herbal medications, and behavioral therapies are being tested in clinical trials and headways have been made in the past decade. The trials included in this review were found by searching “Tourette's Syndrome Treatment” in Pubmed and were selected if they were randomized control trials (RCT) from 2011 until the present. A list of the trials testing pharmacological agents are shown in Table 1.

**Table 1:** Recent pharmacological clinical trials for Tourette syndrome.

Drug	Mechanism	Trial Name	Study Method	Duration	Sample Size	Age of Participants	Primary End Point	Results
Valbenazine (Ingrezza)	Selective VMAT2^1^ inhibitor	T-Forward	RCT	November 2015–December 2016	Phase II (*n* = 124)	18–64 years old	Change in YGTSS from baseline at week 8	Did not meet primary endpoint (*p*-value: 0.18)
		T-Force GREEN	RCT	January 2016–March 2017	Phase II (*n* = 98)	6–17 years old	Change in YGTSS from baseline at week 6	Did not meet primary endpoint
		T-Force Gold	RCT	October 2017–November 2018	Phase II (*n* = 127)	6–17 years old	Change in YGTSS from baseline at week 12	Did not meet primary endpoint
Ecopipam	Selective DRD1^2^ antagonist	NCT02102698	RCT	March 2014–December 2019	Phase II (*n* = 40)	7–17 years old	Change in YGTSS from baseline at day 30	Met primary endpoint
Aripiprazole (Abilify)	DRD2^3^ and 5-HT_1A_^4^ receptor partial agonist and 5-HT_2A_^5^ receptor antagonist	NCT01727700	RCT	July 2011–January 2014	Phase III (*n* = 133)	7–17 years old	Change in YGTSS from baseline at week 8	Met primary endpoint
		NCT00706589	RCT	October 2008–April 2010	Phase III (*n* = 61)	6–18 years old	Change in K-YGTSS from baseline at week 10	Met primary endpoint
Deutetrabenazine (Austedo)	Selective VMAT2 inhibitor	ARTISTS1	RCT	February 2018–November 2019	Phase II/III (*n* = 119)	6–16 years old	Change in YGTSS from baseline at week 12	Did not meet primary endpoint (*p*-value: 0.692)
		ARTISTS2	RCT	May 2018–December 2019	Phase III (*n* = 158)		Change in YGTSS from baseline at week 8	Did not meet primary endpoint (*p*-value: 0.600)

1 VMAT2: Vesicular monoamine transporter 2.

2 DRD1: Dopamine receptor D₁.

3 DRD2: Dopamine receptor D₂.

4 5-HT1A: serotonin 1A receptor.

5 5-HT2A: serotonin 2A receptor.

### 2.6 Behavior therapies

Several recent clinical trials have demonstrated the effectiveness of behavioral therapy in the treatment of patients with TS. A recent RCT comparing CBIT *vs.* control (daily pyridoxine 50 mg and psychoeducation) in patients with TS ages of 6–18 years old showed that the average YGTSS-TTS score of the CBIT arm significantly decreased from a baseline of 19.30 to 10.35 (−46.4%; p < 0.01) at the end of 3 months compared to 17.7 to 14.45 in the non-intervention arm [42]. In a CBIT *vs.* psychoeducation RCT of 61 participants between the ages of 8–15, the YGTSS-TTS decreased at the 3-month follow-up visit for both arms, but more so with CBIT (53.8% compared to 41.3% p < 0.001) [43]. In ERP, patients are trained to suppress any or all tics as they are exposed to greater and greater stimuli (whether it be premonitory urges or environmental factors that elicit tics) for long periods of time [44]. The most recent ERP *vs.* psychoeducation RCT had 221 participants between the ages of 9–17 years old [45]. The treatment response rates were significantly higher in the ERP arm than the psychoeducation arm (47% *vs.* 29%; p = 0.05) [45]. A unique aspect to this study was that it was all done through internet visits and still showed significant improvement in treatment response with ERP. Behavior therapy is already standard of care; however, these trials continue to show the effectiveness of this intervention as a treatment modality for TS.

### 2.7 Pharmacological therapies

#### 2.7.1 Valbenazine

Valbenazine is approved by the FDA to treat tardive dyskinesia and it was granted orphan drug designation for TS by the FDA [46]. Valbenazine is a selective VMAT2 inhibitor, and it was recently tested in three phase II trials for TS.

The first trial, T-Forward (ClinicalTrials.gov, NCT02581865) was a randomized, double-blind, placebo-controlled study consisting of 124 participants with TS between the ages of 18 and 64 [47]. Participants were given either 40 mg or 80 mg doses of valbenazine or placebo for 8 weeks. There was no statistically significant improvement in YGTSS-total tic scores (TTS) for the group that received 40 mg (*p* = 0.433) or the group who received 80 mg (*p* = 0.184) at the end of the 8 weeks [48]. The most common treatment emerging adverse events (TEAEs) were somnolence, fatigue, akathisia, and headache [48].

The second trial, T-Force Green (ClinicalTrials.gov, NCT02679079) was a randomized, double-blind, placebo-controlled study consisting of 98 participants with TS between the ages of 6 and 17 [49]. Participants between the ages of 6 and 11 (children group) were given 10 or 20 mg valbenazine or placebo while those between the ages of 12 and 17 (adolescent group) were given 20 or 40 mg valbenazine or placebo for 6 weeks. There was no statistically significant improvement in YGTSS-TTS for either the children group (*p* = 0.467) or the adolescent group (*p* = 0.888) by the end of the 6 weeks and the study did not reach its primary end point. No serious adverse events were reported and only two participants from the adolescent group discontinued treatment due to TEAEs. The most common TEAEs were headache and somnolence [48].

The final trial, T-Force Gold (ClinicalTrials.gov, NCT03325010) was a randomized, double-blind, placebo-controlled study consisting of 127 participants between the ages of 6 and 17 with moderate to severe TS [50]. Participants were given either 20 or 40 mg of valbenazine or the placebo as the initial dose (for subjects <50 kg or >50 kg, respectively) and the dose was raised to a maximum of 60 or 80 mg (for subjects <50 kg or >50 kg, respectively) over the course of 6 weeks. At the end of the 6th week, the subjects continued their maximum dosage for 6 more weeks. There was no significant reduction in YGTSS -TTS at the end of 12 weeks (*p* = 0.177) and 8 participants discontinued use of valbenazine due to TEAEs such as headache and somnolence [48].

#### 2.7.2 Ecopipam

Ecopipam is a selective D1 receptor antagonist that received a Fast Track designation from the FDA for TS [51]. A randomized, double-blind, placebo-controlled phase II clinical trial (ClinicalTrials.gov, NCT02102698) was conducted consisting of 40 participants with TS between the ages of 7 and 17 [52]. Participants took ecopipam at the dose of 12.5 mg, and the dose was subsequently titrated up based on weight (50 mg for children <34 kg and 100 mg for children >34 kg). This trial had a cross-over design. Participants were randomly assigned to be treated first with ecopipam then placebo or vice versa. Ecopipam performed statistically better than placebo in reducing YGTSS-TTS (*p* = 0.033), reaching its primary endpoint at the end of its 30 day trial [52,53]. Two participants in the ecopipam group withdrew due to insomnia and a foot fracture, but both were deemed unrelated to the drug by the investigator. The most common adverse effects were headaches, somnolence, insomnia, nausea, and vomiting [53].

#### 2.7.3 Aripiprazole

Aripiprazole is a D2 and 5-HT_1A_ receptor partial agonist and 5-HT_2A_ receptor antagonist that is FDA-approved for autism spectrum disorder (ASD), schizophrenia, and bipolar disorder [54]. Aripiprazole has been used for treating TS off label. Two randomized, double-blind, placebo-controlled clinical trials were conducted to assess the efficacy and safety of aripiprazole use for TS [55,56]. Both studies met their primary end points and are discussed in detail in the following paragraphs.

A randomized, double-blind, placebo-controlled Phase III trial to test the efficacy of aripiprazole on tics (ClinicalTrials.gov, NCT01727700) by assessing the change in YGTSS-TTS at baseline compared to the end of 8 weeks [55]. This study consisted of 133 participants with TS between the ages of 7–17. Participants were randomized to either a low or high dose of aripiprazole based on weight (5 mg/day if < 50 kg; 10 mg/day if ≥ 50 kg for low dose) and (10 mg/day if < 50 kg; 20 mg/day if ≥ 50 kg for high dose), or a placebo daily. In this study, 69% (29/42) of patients in the low-dose group and 74% (26/35) of patients in the high-dose group had statistically significant improvements in Clinical Global Impression-TS scale compared to 38% (16/42) in the placebo group. The change in YGTSS-TTS from baseline, which is the primary end point, at the end of 8 weeks was also statistically significant with the high dose group (*p* < 0.0001) and the low dose group (*p* = 0.002), when compared to the placebo group [55]. The most common adverse effects in this study were sedation, somnolence, and fatigue [55].

Another randomized, double-blind, placebo-controlled Phase III trial with a similar design (ClinicalTrials.gov, NCT00706589) consisted of 61 participants between the ages of 6–18 [56]. Participants were given either a mean dose 11.0 mg of aripiprazole (starting dose being 2–2.5 mg, titrated every 1–2 weeks for tolerability, up to 20 mg) or a placebo daily. Those who received aripiprazole had significant reductions in YGTSS-TTS compared to placebo (*p* = 0.0196) [56].

#### 2.7.4 Deutetrabenazine

Deutetrabenazine, the deuterated form of tetrabenazine, has a longer half-life compared to tetrabenazine [57]. Deutetrabenazine is also a selective VMAT2 inhibitor [58]. Two clinical trials, ARTISTS1 (phase II/III) and ARTISTS2 (phase III), were conducted to assess the efficacy and safety in children with TS [59,60].

The first trial, ARTISTS1 (ClinicalTrials.gov, NCT03452943) was a phase II/III randomized, double-blind, placebo-controlled study consisting of 119 participants with TS between the ages of 6 and 16 [59]. Participants were given an initial dose of deutetrabenazine at 6 mg/day and the subsequent doses were titrated based on body weight and cytochrome P450 2D6 (CYP2D6) status. There was no significant change in YGTSS-TTS (*p* = 0.690) from baseline at the end of 12 weeks. Thus the study did not meet its primary endpoint [61]. No serious adverse events were reported and the most common TEAEs were fatigue, weight increase, and headache [61].

The second trial, ARTISTS2 (ClinicalTrials.gov, NCT03571256) was a phase III randomized, double-blind, placebo-controlled study consisting of 158 participants with TS between the ages of 6 and 16 [60]. Participants were given either a low (up to 36 mg) or high (up to 48 mg) dose of deutetrabenazine or placebo. Both the high dose and low dose group did not reach the primary endpoint to demonstrate reductions in YGTSS-TTS (*p* = 0.600 and *p* = 0.474 respectively) [62]. The most common TEAEs were somnolence, headache, and nasopharyngitis [62].

### 2.8 Alternative therapies

Alternative therapies like Chinese traditional medicine (CTM) are shown to have some benefit for the treatment of TS although their efficacy is still up for debate. A metanalysis of the 26 trials that utilized YGTSS to assess tic severity found that those who used CTM showed significant improvement in YGTSS-TTS compared to those in the control groups (SMD = −0:21, 95% CI: −0.29 to −0.14, I2 = 12:30%) [63]. The 5-ling granule (5-LGr) and Ningdong granule are common CTM used to treat TS in China. They are both acknowledged by the European clinical guidelines, but are not recommended for treatment [64]. The only RCT for the 5-LGr had 603 participants (between the ages of 5–18 years old) who were randomly assigned to either the placebo, tiapride (200–400 mg/day), or 5-LGr arm (15–22.5 g/day). When compared to the placebo, the 5-LGr significantly decreased the participants’ YGTSS-TTS (*p* < 0.001) by the end of 8 weeks [65]. There is more research for the Ningdong granule than the 5-Lgr with both clinical trials and animal models [66,67]. In one RCT for the Ningdong granule, 68 participants were randomly assigned to the Ningdong granule arm (1 g/kg per day) or the placebo arm. By the end of 8 weeks, the Ningdong granule arm had a significant reduction in YGTSS-TTS from a baseline of 23.00 to 13.48 (−41.39%) compared to placebo 22.42 to 20.00 (−10.79%) (p < 0.001) [66]. CTM has shown promising results for the treatment of TS, but more studies are needed.

### 2.9 Deep brain stimulation (DBS)

DBS is generally a treatment reserved for individuals with severe tics due to the invasive nature of the procedure [68]. Electrodes are implanted in specific locations of the brain to generate electric currents to modulate neuron firing. Bilateral lead placement is generally preferred over unilateral [69]. According to the European clinical guidelines for TS, DBS should only be performed on adults if the patient does not respond to behavioral therapy and multiple pharmacotherapies with tic symptoms persisting for at least 5 years and at least 1 year of severe symptoms (YGTSS TS of at least 35) [64,69]. It is not readily available for all patients because it can only be done at specialized centers so there are few randomized-control studies assessing their efficacy. Trials are still being done to determine the best placement for the electrodes to maximize tic reduction. The most commonly used sites are the globus pallidus interna (GPi) and the thalamus (Centromedian-Parafascicular Complex (CM-Pf)) [70].

#### 2.9.1 Globus pallidus internus (GPi)

The most common site of implantation is the GPi. The GPi is part of the basal ganglia circuit, which is thought to play a critical role in TS [71,72]. All nine studies with bilateral GPi stimulation have reported improvements in the YGTSS-TTS with 5 of the studies showing improvement by at least 50% (Table 2). There was a total of 83 participants with TS with ages ranging from 15 to 55 years old in these studies. In one study, with a pool of 15 TS patients and follow-up of 17–82 months, a 38.2% overall improvement in the YGTSS-TTS was reported [73]. Another study of 13 TS patients with a follow-up range of 13–80 months reported an improvement of YGTSS-TTS by 52.1% [74]. There was one case where the participant experienced anxiety and depression that lead to electrode removal [74]. In one case study, the participant experienced impairment in his ability to use his hand, particularly with alternating supination and pronation movements [75].

**Table 2:** Recent deep brain stimulation clinical trials.

Target Site	Number of Participants	Age Range	Frequency (Hz)	Volt (V)	Pulse width (μs)	Change in total YGTSS	Adverse Effects
Bilateral amGPi [73]	15	N/A	80–130	1–4.2	60–240	88.1 to 53.9 (−38.2%)	Some patients experienced nausea, dizziness, weight gain, etc.
Bilateral GPi [74]	13	16–34	185	3.6	120	63.5 to 30.4 (−52.1%)	One patient experienced anxiety and two experienced agitation. One experienced constant depression and tiredness that lead to lead removal. One patient had pyosis. One had a chest infection due to hardware.
Bilateral GPi [75]	1	27	185	2	60–150	83.0 to 44.0 (−47.0%)	The patient experienced mild transient fatigue but had impairment in left extremities (unable to perform alternating pronation and supination movements).
Bilateral STN and GPi [125]	4	20–28	135–145	2.35–3.30	2–70	74.7 to 41.0 (−45.1%)	One participant withdrew from the trial due to lack of improvement.
Bilateral GPi [126]	15	24–55	125–180	0.8–4.0	60–180	87.9 to 68.3 (−15.3%)	Two patients had hardware infections. One experienced a hypomania episode.
Bilateral GPi [127]	19	19–57	130	2.5–4	60–150	75.3 to 45.0 (-40.2%)	Four patients had hardware infections. One patient experienced increased tic severity. Two patients experienced nausea and vertigo. Two patients had sleeping disorders. Two patients had falls. Three patients experienced dysarthria. One patient experienced dyskinesia-like movements. Two patients experienced weight-gain.
Bilateral amGPi [128]	11	18–50	130–160	3.0–5.0	60–120	84.5 to 42.3 (−51.0%)	None
Bilateral GPi [129]	15	34–54	100–180	2.2–5.6	180–360	42.2 to 12.8 (−69.7%)	One patient had a coagulase-negative staphylococcus infection. Two patients experienced apathy. One patient experienced weight loss and stimulation-related agitation.
Bilateral amGPi [130]	1	15	130	3.0–3.5	90–120	81.0 to 32.0 (−60.5%)	None
Bilateral GPi [131]	2	22–41	130–160	2.8–3.5	90	51.0 to 22.5 (−55.9%)	None
Bilateral CM-Pfc [78]	11	17–46	N/A	N/A	N/A	85.4 to 41.0 (−54.0%)	One patient experienced recurrent tension headache, worsening of pre- existing tremor, and transient blurring of vision. One patient experienced dizziness. One patient experienced, mild paresthesia. One patient had a hardware infection. One patient experienced reoccurring suicidal thoughts. One experienced involuntary jaw movements.
Bilateral CM-Pf [81]	1	28	180	N/A	87	87.0 to 27.0 (−69.0%)	None
Bilateral CM-Pfc [79]	18	17–47	120–130	2.5–4.0	90–210	80.8 to 28.6 (-64.6%)	Most patients experienced vertigo, blurring of vision and abdominal discomfort. One patient had upward ocular deviation.
Bilateral CM-Pfc [82]	3	17–35	107–130	2.5–4.1	90–120	81.0 to 25.0 (−70.0%)	None
Bilateral CM-Pfc [80]	5	18–34	130–185	3.5–3.6	90–210	YGTSS Tic Severity 37.2 to 28.2 (−24.2%)	Four participants experienced decline in verbal fluency. One participant experienced increased depression and anxiety.
Bilateral CM-Pfc [83]	1	27	125	0.9	120	YGTSS Tic Severity (−47.9%)	None
Bilateral CM-Pfc [84]	5	28–39	125	0.3–1.1	80–320	(-30.0%)	None

#### 2.9.2 Centromedian-parafascicular complex (CM-Pfc)

The centromedian-parafascicular complex (CM-Pfc) is also a common site for DBS electrode placement. Located within the intralaminar nuclei of the thalamus, the CM-Pfc plays a role in arousal, sensory awareness, pain control, behavior and cognition [76]. Stimulation of the CM-Pfc can possibly regulate motor, associative, and limbic circuits [77]. All seven studies assessing bilateral CM-Pfc stimulation for TS have reported improvements in the YGTSS-TTS with 4 of the studies showing improvement by over 50% [78–84] (Table 2). There was a total of 44 participants with ages ranging from 17 to 47 years old. In one study with follow-up ranging from 3 to 18 months, all of the 18 participants reported an improvement in YGTSS (mean YGTSS-TTS from 80.833 to 28.556; *p < 0.001*) [79]. Another study with a pool of 11 TS patients with a follow-up range of 2–91 months (averaging 26 months) reported a 54.0% improvement in YGTSS-TTS [78]. With regards to adverse events, there were reports of blurred vision in two of the studies [78,79]. Two participants in two separate studies reported increased depression [80] or recurring suicidal thoughts.

#### 2.9.3 Location comparisons

Aside from case studies and DBS vs. sham trials, there have been RCTs comparing different locations for DBS, particularly the thalamus and the globus pallidus. In a RCT by Houeto et al., a 36-year-old woman had electrodes placed in both the bilateral GPi and the bilateral CM-Pfc [85]. Stimulation parameters were 130 Hz for frequency, 60 μs for pulse width, and 1.5 V for voltage. When the bilateral GPi were stimulated the patient was able to control her tics but she experienced increased nausea, hypotonia, and anxiety. Her YGTSS-TTS changed from a baseline of 84 to 29 (−65.5%). When the bilateral CM-Pfc were stimulated, self-injurious behavior completely resolved, and the tics improved. Her YGTSS-TTS changed from a baseline of 84 to 30 (−64.3%). When both the bilateral GPi and the bilateral CM-Pfc were stimulated, self-injurious behavior completely resolved, and her YGTSS-TTS changed from a baseline of 84 to 34 (−59.5%). In a similar RCT by Welter et al., three patients, between the ages of 30 and 36 years old, had electrodes implanted in both the bilateral GPi and the bilateral CM-Pfc [86]. Stimulation parameters were 130 Hz for frequency and 60 μs for pulse width (the voltage was unspecified). When the bilateral GPi were stimulated there was an average change of −78.3% in YGTSS-TTS. When the bilateral CM-Pfc were stimulated there was an average change of −44.7% in YGTSS-TTS. When both the bilateral GPi and the bilateral CM-Pfc were stimulated there was an average change of −59.7% in YGTSS-TTS. No adverse events were reported. In a slightly different RCT by Müller-Vahl et al., ten patients between the ages of 18 and 47 years old had electrodes implanted in both the bilateral GPi and the bilateral centromedian-ventro-oral internus (CM-Voi) [87]. Stimulation parameters were 130 Hz for frequency, 210 μs for pulse width, and a voltage range of 2.5–4 V for GPi and a voltage range of 1.8–3 for CM-Voi. When the bilateral GPi were stimulated there was an average change of −14.8% in YGTSS-TTS (from 39.11 to 33.33). When the bilateral CM-Voi were stimulated there was an average change of −5.1% in YGTSS-TTS (from 39.11 to 37.11). Some of the patients experienced tremors, dystonic movements of hands, dysphoric feeling, paresthesia, headaches, and dizziness. In summary, the GPi could be an appealing DBS targets for TS while other targets should also be considered. Large sample size RCTs are needed to determine the optimal DBS targets for TS.

### 2.10 Repetitive transcranial magnetic stimulation (rTMS)

Only one RCT has been published looking into the efficacy of rTMS in people with TS. In this study, 20 adults with severe TS were divided into 2 groups, both of which had 15 sessions (1-Hz; 30 min; 1800 pulses per day) of either active or sham rTMS over the supplementary motor area (SMA) [88]. YGTSS-TTS was assessed after three weeks and those receiving active treatment had a 17.3% reduction compared to sham who had a 13.2% reduction, but this was not significant (p = 0.27). There was an open label extension for 3 weeks involving 7 participants who were initially randomized to active treatment did result in a 29.7% reduction of tic severity, which was statistically significant (p = 0.04) [88]. A larger double blind RCT is currently underway in Alberta, Canada recruiting 50 children to either active rTMS plus CBIT or to sham rTMS plus CBIT targeting the SMA with the primary outcome measure as change from of TS severity as measured by the YGTSS [89].

### 2.11 Recent advances in neuroimaging

Novel therapy development for movement disorders often hinges on the knowledge of the pathophysiology as well as circuit connections. Along this line, magnetic resonance imaging (MRI) is a powerful tool to understand structural differences in the brains of individuals with TS, and several structural MRI studies have found alterations in the volume of different brain structures in TS patients.

In one MRI study, which included 154 children and adults with TS and 130 control subjects, the volumes of the caudate and lenticular nucleus for those with TS were smaller than the control subjects [90]. Another study found that the volume of the caudate nucleus can be a predictor of tic severity in adulthood in children with TS [91]. The participants’ total childhood caudate volume correlated inversely with their YGTSS in late adolescence [91]. However, there are previous studies that do not show this pattern. One study of 37 children with TS and 18 controls found no significant differences in the size of basal ganglia (such as the putamen, caudate nucleus, and globus pallidus) between those with TS and controls [92].

The thalamus is another brain region with possible structural changes in TS. A cross-sectional study of 149 affected individuals and 134 controls found that thalamic volumes of TS patients were larger than those of controls, but there was no correlation between tic severity and the volume of the thalamus [93]. In another study, 18 TS boys who did not receive treatment were compared to 15 unaffected boys, and the boys with TS were found to have a larger left thalamus, but no significant difference in the size of the right thalamus compared to controls [94]. Imaging of thalamic nuclei as well as the basal ganglia has therapeutic implications for individuals with TS undergoing DBS. It is thought that DBS helps patients with TS due to the stimulation of networks rather than local brain regions. By using tractography, therapeutic networks are being identified to improve tics. In a study of 66 patients who underwent DBS (34 with GPi implantation and 32 with centromedial thalamic implantation), those with GPi stimulation were found to have improvement in tics through the limbic and associative networks, while those with centromedial thalamic stimulation had improvement mediated through the sensorimotor and parietal-temporal-occipital networks [95]. This information can help better localize where to implant DBS electrodes to optimize therapeutic benefit.

Studies have been conducted to see if there are changes in cortical gray matter volume in individuals with TS. One voxel-based morphometry (VBM) study comparing 40 adults with TS to 40 healthy individuals found no differences in intracranial volume between individuals with TS and controls [96]. Individuals with TS had reduced gray matter volume in the medial orbitofrontal, rostral cingulate, ventrolateral prefrontal cortex and operculum, but greater gray matter volume in the putamen. There was no correlation between gray matter volume and tic severity [96]. In a larger whole brain MRI study, 103 TS children were matched with 103 controls by age, sex, and handedness. Those with TS had reduced white matter volume in orbital and medial prefrontal cortex, but greater gray matter volume in the posterior thalamus, hypothalamus, and midbrain, than those without TS [97].

The corpus callosum is the communication network between the two halves of the cerebral hemispheres and network changes have been seen in patients with TS. One study using diffusion tensor imaging (DTI) compared 20 TS boys with 20 age and gender-matched controls and found reduced corpus callosum connectivity in individuals with TS though there was no correlation with tic severity [98]. A MRI-DTI study on monozygotic twins discordant of TS also showed decreased corpus collosum connectivity in the affected twin [99]. Regarding the size of the corpus collosum, there have been contradicting studies. One found that there was a larger size of the corpus callosum in individuals with TS [100], and another study found no significant differences in the size of the corpus callosum in TS patients [101]. It is unclear whether the discrepancies between studies is due to patient selection or analysis methodology.

The limbic system has also been investigated in TS. One study has found that while the hippocampus and amygdala volumes are larger in children with TS, the volumes are smaller in adults with TS when compared to age-matched controls [102]. This suggests a dynamic modulation throughout neurodevelopment.

Functional MRI (fMRI) can also help to elucidate the pathophysiology of TS. An early fMRI study found an increase in the activation of the sensorimotor cortex and supplementary motor areas of individuals with TS compared to those without TS during finger-tapping [103]. However, increased activation in these brain regions in individuals with TS was not found in another fMRI study [104]. One study used fMRI as a feedback tool to treat TS. This small, randomized trial was recently conducted using real-time fMRI as neurofeedback intervention. In this group of 21 individuals with TS between the ages of 11–19, participants with neurofeedback had a greater reduction in YGTSS-TTS (3.8 point reduction) compared to those without neurofeedback *(p* < 0.05) [105]. This study provides a proof-of-principle for neurofeedback in TS.

We are just beginning to understand the structural changes in the brains of individuals with TS and studies so far have demonstrated varied results, which are at times conflicting. TS is likely to be a heterogeneous disorder and brain structural alterations in TS could have patterns specific to age (children *vs.* adults), gender (male *vs.* female), tic severity and neuropsychiatric comorbidities. These factors should be taken into consideration in future TS neuroimaging studies. In addition, neuroimaging studies may be able to help to stratify heterogeneous TS population. Techniques such as fMRI and tractography can further aid monitoring brain network changes and precisely target TS brain networks via DBS, respectively.

### 2.12 Electrophysiology in Tourette syndrome

Electrophysiology, particularly the use of electroencephalography (EEG), in patients with TS is a tool that can be used to help understand the neurophysiologic basis of TS and is helping to guide experimental non-invasive treatments. Studies with small sample sizes have been done in children with TS showing that they have distinct EEG patterns compared to healthy controls. One study looked at monozygotic twins with TS and found the more severely affected twin to have more fronto-central theta activity [106]. Another study has also shown that there is reduced long range connectivity between the frontal and temporal/occipital/parietal lobes in patients with TS compared to healthy controls, which mirrors results in fMRI studies [107,108]. It is hypothesized that dysrhythmic thalamo-cortical oscillations may lead to a loss of neuronal control over movements and lead to tics [109]. Therapies are being targeted to improve the rhythmicity of the oscillations using tools such as neurofeedback to train the brain to gain control over neuronal processes and behavior [110]. Repetitive transcranial magnetic stimulation (rTMS) as well as transcranial direct current stimulation (tDCS) also use electrophysiological information to guide treatment. rTMS was shown in a small double blind RCT to improve tic severity [88]. Non-invasive therapies that harness electrophysiologic changes in TS hold promise as a future treatment for those with TS.

### 2.13 Recent advances in genetics

Although most cases of TS are sporadic, a few genetic family studies have found that TS may have a degree heritability, especially amongst first degree relatives. TS is generally not a monogenetic disease; rather, poly-genetic contributions are likely. A study using the Swedish National Patient Registry has found that first-degree relatives had a significantly higher chance of developing tic disorders (odds ratio [OR], 18.69; 95% CI, 14.53–24.05) (despite different living environments) compared to second-degree (OR, 4.58; 95% CI, 3.22–6.52) or third-degree (OR, 3.07; 95% CI, 2.08–4.51) relatives [111]. Within first-degree relatives, full siblings with 50% genetic similarity, (OR, 17.68; 95% CI, 12.90–24.23) had a much higher risk than half siblings with 25% genetic similarity, (OR, 4.41; 95% CI, 2.24–8.67) despite similar living environments [111]. Although there is high heritability, no distinct gene has been identified as causing TS. On the other hand, several recent genetic studies have identified new genes as potential therapeutic targets.

#### 2.13.1 SLITRK1

Slit and Trk-like 1 (*SLITRK1*) on chromosome 13q31.1 was among the first major breakthroughs for TS genetic research [112]. The first proband identified was the only one in the pedigree affected with TS and is the only one with a de novo chromosome 13 inversion in proximity to the *SLITRK1* gene. *SLTRK1* is expressed in the striatum, globus pallidus, thalamus, and subthalamus of the fetal brain, areas implicated for TS [112,113]. When cultured, wild-type human *SLITRK1* cortical pyramidal dendrites were significantly longer than dendrites with a *SLITRK1* frameshift mutation. This suggests the frameshift is a loss of function mutation, which may hinder dendritic growth [112]. However, these mutations are only present in a small subset of those affected with TS and the exact pathogenesis of the mutation is still unclear.

#### 2.13.2 l-Histidine decarboxylase (HDC)

W317X nonsense mutations (missing 316 amino acids) of the *HDC* gene on chromosome 15q21-q22 was identified in a genome wide analysis of two generations of a family [114]. The 3.4-centimorgan (cM) segment of chromosome 15 contained the W317X mutation, a terminating mutation of exon 9 of HDC [114]. HDC is an enzyme crucial in converting histidine into histamine suggesting the possibility of histamine disruption playing a role in TS. In a genetic study, the father and his 8 children who were all diagnosed with TS had these mutations while the mother and her extended family did not have the mutation, nor did they have any history of TS or other tic disorder [115]. *HDC* Knockout mice exhibit tic-like behavior, induced by psychostimulants like d-amphetamine, whereas intracerebroventricular infusion of histamine can suppress these behaviors [116], demonstrating the importance of histaminergic neurotransmitters in tics.

#### 2.13.3 PNKD

A heterozygous nonsense mutation in the *PNKD* gene (stands for Paroxysmal Nonkinesigenic Dyskinesia) was found in a genetic family study. In the three-generation TS multiplex family, all the affected individuals of the family shared the heterozygous nonsense mutation (chr2: 219204814 C/T) [117]. This genetic mutation results in reduced transcript and protein levels, and also mis-localization of the PNKD long isoform protein [117]. It is hypothesized that there is a PNKD protein insufficiency during brain development in TS patients.

#### 2.13.4 FLT3

*FLT3* encodes fms-like tyrosine kinase, a receptor tyrosine kinase. A recent genome-wide association study (GWAS) identified that *FLT3* is linked to TS [118]. The FLT3 ligand is associated with the development and activation of immune cells, such as dendritic cells and natural killer cells, since it induces monocyte proliferation [119]. One cross-sectional study found that the number of monocytes is higher in those with TS compared to controls [120]. This link between the increased expression of *FLT3* and increased levels of monocytes may suggest that the immune system plays a role in the pathogenesis of TS.

#### 2.13.5 Other genes

A few other tentative candidates for TS risk alleles have been found in association studies, including *NRXN1*, on chromosome 2p16 and *CNTN6,* on chromosome 3p26 [121]. In one association study, five unrelated individuals with a de novo mutation of *ASH1L* have been identified using whole-exome sequencing [122]. In addition, mouse models of *ASH1L*^+/−^ exhibited tic-like jerky movements and they responded to haloperidol [122], further supporting the role of *ASH1L* in tics. *CELSR3*, which encodes for a cadherin receptor and is important for cell polarity, has also been found to be associated with TS [123].

Several genetic mutations and variants have been found to be associated with TS, and mouse models deficient in *HDC* and *ASH1L* have been created which were found to recapitulate some of the tic features of TS [116,122]. These studies are instrumental in our understanding of the pathological mechanisms of TS and the mouse models with these genetic mutations could be a novel platform for therapeutic development to treat tics.

## 3 Conclusion

TS is a disorder that can severely disrupt activities of daily living and are associated with anxiety, depression and social stigmatization due to the disruptive nature of tics. The treatment options for TS remain limited and emerging pharmacological therapies like ecopipam are still being tested. DBS has been used to treat medication refractory TS, but further studies are needed to identify optimal targets. To determine the definite safety and efficacy of DBS for TS, randomized controlled trials with blinded assessments and larger sample sizes are needed. Studies investigating neuronal firing patterns can use DBS electrodes with recording capabilities to provide further insight into the pathophysiology of TS. In addition, recent advances in genetics and neuroimaging have improved our understanding of TS pathophysiology and anatomic localization. Improved understanding of the disease using genetic tests as well as biomarkers will hopefully drive future therapeutic development to provide treatment choices tailored for each TS patient. With the need for more trials and studies, patient involvement is especially important for larger scale research [124].

## Author contribution statement

All authors listed have significantly contributed to the development and the writing of this article.

## Funding statement

Sheng-Han Kuo was supported NINDS [R01NS104423; R01NS118179; R01NS124854].

## Data availability statement

Data included in article/supp. material/referenced in article.

## Declaration of interest’s statement

The authors declare no competing interests.
